RETRACTED

# Overexpressed C14orf166 associates with disease progression and poor prognosis in non-small-cell lung cancer

**DOI:** 10.1042/BSR20180479

**Published:** 2018-09-14

**Authors:** Yan-Wu Zhou, Rong Li, Chao-Jun Duan, Yang Gao, Yuan-Da Cheng, Chun-Fang Zhang

**Affiliations:** 1 Department of Thoracic Surgery, Xiangya Hospital, Central South University, Changsha 410008, Hunan Province, China; 2 Department of Gastroenterology, Xiangya Third Hospital, Central South University, Changsha 410013, Hunan Province, China; 3 Institute of Medical Science, Xiangya Hospital, Central South University, Changsha 410008, Hunan Province, China

**Keywords:** C14orf166, Clinicopathology, Disease progression, Non-small cell lung cancer, Prognosis

## Abstract

Chromosome 14 ORF 166 (C14orf166), a protein involved in the regulation of RNA transcription and translation, has been reported to possess the potency to promote tumorigenesis; however, the role of C14orf166 in non-small-cell lung cancer (NSCLC) remains unknown. The purpose of the present study was to assess C14orf166 expression and its clinical significance in NSCLC. Immunohistochemical staining, quantitative real-time PCR (qRT-PCR), and Western blotting were used to detect the C14orf166 protein and mRNA expression levels in NSCLC tissues compared with adjacent normal tissues, as well as in NSCLC cells lines compared with normal human bronchial epithelial cells (HBE). Then, the correlations between the C14orf166 expression levels and the clinicopathological features of NSCLC were analyzed. Additionally, the Cox proportional hazard model was used to evaluate the prognostic significance of C14orf166. We found that C14orf166 expression increased in carcinoma tissues compared with their adjacent normal tissues at the protein (*P*<0.001) and mRNA levels (*P*<0.001). High expression of C14orf166 was significantly associated with the T stage (*P*=0.006), lymph node metastasis (*P*=0.001), advanced TNM stage (*P*<0.001), and chemotherapy (*P*<0.001). Moreover, according to the survival analysis, patients with overexpressed C14orf166 were inclined to experience a shorter overall survival and disease-free survival time (*P*<0.001). Multivariate COX analysis implied that C14orf166 was an independent prognostic biomarker. Taken together, our findings indicate that the overexpression of C14orf166 may contribute to the disease progression of NSCLC, represent a novel prognostic predictor and help high-risk patients make better decisions for subsequent therapy.

## Introduction

Lung cancer is a well-known malignant disease, with the highest morbidity and mortality worldwide, moreover, nearly 40% patients were found with metastatic lesions at diagnosis [1,2]. Non-small-cell lung cancer (NSCLC) accounts for approximately 80% of total lung cancer pathological types, and it mainly consists of adenocarcinoma and squamous cell carcinoma [3]. Surgery is the main treatment for lung cancer, and adjuvant chemotherapy has gradually become common in patients with proper indications post-operation. Cisplatin is generally recommended for the treatment of advanced NSCLC; however, the efficacy of cisplatin is increasingly unsatisfactory because of the emergence of drug resistance, resulting in a 5-year survival rate that is still less than 15% [4,5]. Further investigations to explore the underlying mechanisms of NSCLC and to find novel biomarkers and therapeutic targets are needed to change this clinical dilemma.

RETRACTED

Chromosome 14 ORF 166 (C14orf166), also known as CGI-99, CGI99, CLE, CLE7, LCRP369, or RLLM1, is a 28-kDa protein located in the nucleus and in the cytoplasm, while its conserved gene is located on chromosome 14 at 14q22.1 [6]. As a component of nuclear and cytoplasmic protein complexes, C14orf166 was first found to be involved in viral RNA replication and transcriptional activation during influenza A virus infection through stimulating host RNAP II and viral RNA polymerase activities [7,8]. Then, C14orf166 was reported to act as a shuttling protein that helps substances involved in RNA metabolism shuttle between the nuclei and the cytoplasm. Furthermore, C14orf166 interacts with RNAP II and regulates RNA transcription directly, indicating a vital role of C14orf166 in cell growth and organ development [9]. It has been demonstrated that C14orf166 is responsible for nearly half of the mRNA translation participating in the cell cycle; therefore, the deletion of C14orf166 induces a loss of major cellular function [10]. In addition to its role in RNA metabolism as a binding partner of JAK2, C14orf166 is also involved in signal transduction, specifically through the signal transducer and activator of transcription 3 (STAT3 pathway), which is thought to regulate part of the downstream oncogenes shared by β-catenin [11]. It has been reported that the excessive activation of STAT3 participates in the pathogenesis of considerable tumors [12–14]. In esophagus carcinoma cells, overexpressed C14orf166 has been reported to activate the abnormal JAK2/STAT3 signaling pathway by acting as a JH2-interacting protein, which induces excessive function, initiating carcinogenesis [15–17]. Additionally, along with our previous research in esophagus squamous cell carcinoma [18], C14orf166 is found to be overexpressed in several tumor tissues [19–22]; however, the role of C14orf166 in NSCLC is unknown, and this present study aims to clarify this potency.

RETRACTED

In the present study, we compared the expression of C14orf166 in cancerous tissues and cells with their respective normal controls at the protein and mRNA levels with immunohistochemistry (IHC), Western blot analysis, and quantitative real-time PCR (qRT-PCR). Furthermore, we explored the relationship between C14orf166 expression and the clinicopathological features and prognosis in NSCLC patients (NSCLCs).

## Materials and methods

### Ethical statement

Written informed consent was obtained from all the participants, and the study protocol was approved by the ethics committee of Xiangya Hospital, Central South University.

### Clinical samples and cell lines

NSCLC tissues and paired normal lung tissues were obtained from 125 patients (median age: 60 years, range: 39–76 years) who underwent lung resection between July 2010 and December 2012 at Xiangya Hospital in Central South University. There were 32 women and 93 men enrolled in our present study. None of the patients had a history of previous malignancies, chemotherapy, or radiotherapy before sampling. The clinical and pathological data were complete and reliable. Tumor differentiation and staging was classified according to the eighth edition of TNM classification of UICC. One part of each sample was immediately snap-frozen in liquid nitrogen and was stored at −80°C for RNA and protein extraction. The other part of each sample was fixed in 10% neutral PB-buffered formalin (pH 7.4) for IHC. All the tissues were histologically confirmed by two pathologists.

The subjects were followed up every 3 months during the first post-operative year and at least 6 months afterward for survival and recurrence inquiry until death or until the end of the investigation.

Human NSCLC cell lines (A549, PC-9, and HTB182) and normal human bronchial epithelial cells (HBE) were obtained from Chinese Academy of Science Cell Bank (Shanghai, China). The cells were cultured and maintained in RPMI 1640 supplemented with 10% FBS),100 U/ml penicillin and 100 ug/ml streptomycin in a humidified incubator with 5% CO_2_ at a temperature of 37°C. All the culture materials were purchased from Gibco, U.S.A.

### qRT-PCR

We followed the specific experimental procedure details previously described [17]. The total RNA was extracted from the tissues or cells by using TRIzol (Invitrogen, U.S.A.) according to the manufacturer’s protocol. After treatment with DNA-free (Ambion, U.S.A.) to remove the chromosomal DNA, the cDNA was synthesized using the Reverse Transcription Kit (Promega, U.S.A.) and was stored at −20°C until use. The mRNA expression levels of C14orf166 and β-actin were determined by qRT-PCR using the ABI PRISM 7500 sequence detector system (Applied Biosystems, U.S.A.). The primer sequences were sense/antisense: C14orf166: 5′-TGCATTGTCAGCAGTTTTTGA-3′/5′-TGACTGGCTTCTTGGTTTAGC-3′; and β-actin: 5′-GCACCACACCTTCTACAATGAG-3′/5′-GATAGCACAGCCTGGATAGCA-3′. The mRNA expression levels of the target genes were normalized to the β-actin signal. All the reactions were performed in triplicate using 20 μl samples containing 50 ng of cDNA. The reaction protocol involved heating for 10 min at 95°C, followed by 40 cycles of amplification (15 s at 95°C and 1 min at 60°C). The data were analyzed using the ABI PRISM 7500 Sequence Detection software. The relative expression of C14orf166 was described as 2^−ΔΔ*C*^_t_.

RETRACTED

### Western blotting analysis

The cultured cells or tissues were harvested and lysed with RIPA lysis buffer (Beyotime, China) for 30 min on ice. After centrifugation at 12000 ***g*** for 20 min, the concentration of the proteins was measured using Bradford’s reagent (Bio-Rad Laboratories, U.S.A.). The protein samples were denatured by boiling for 10 min and were loaded on to SDS/PAGE (10% gel) for electrophoresis. The proteins were transferred on to a PVDF membrane (Millipore, U.S.A.), which was then incubated in the blocking solution (5% FBS) at room temperature for 1 h. The anti-C14orf166 (1:1000 (1 mg/ml), Proteintech, U.S.A.) was added into blocking solution and incubated at 4°C overnight. The membranes were subsequently incubated with HRP-labeled goat anti-rabbit IgG for 1.5 h at room temperature. Protein expression was normalized against GAPDH expression (1:1000, RD, U.S.A.). Bands were visualized by employing the BeyoECL Plus Detection System (Beyotime, China) and Bio-Rad Image Lab Software (CA, U.S.A.).

### Immunohistochemical staining

The rapid PV two-step staining method with the following specifications was used: paraffin slice thickness of 5 μm, slices heated at 65°C for 60 min, dewaxed in xylene, rehydrated in an increasing diluted ethanol series, high-temperature antigen retrieval via microwave in 0.1 M citrate solution (pH 6.0) for 10 min, 3% H_2_O_2_ incubated at room temperature for 20 min, goat serum at room temperature incubated for 20 min, incubated anti-C14orf166 rabbit polyclonal antibody (1:100 (10 mg/ml), Proteintech, U.S.A.) at 4°C overnight, rewarmed the next day, incubated with the second anti-rabbit antibody at room temperature for 20 min, DAB coloration, Hematoxylin were mounted, and then microscopic examination. Results interpretation method: IHC was scored independently by two pathologists without knowledge of patient information, and any discrepancy was solved by consensus review. The score of immunoreactivity was performed by calculating the extent and intensity of staining positivity of cells in a semiquantitative manner. As described previously [23], the standards for evaluation included as following: positive stain intensity (0, negative; 1, weak; 2, moderate; 3, strong) and proportion of positive areas (≤10% = 1; 10–50% = 2; ≥50% = 3). The staining score was the multiplication of the previous two scores. Five high power fields in each specimen were selected randomly, and the final score is the average of the five scores. The samples were classified as weak staining when the final scores were 0–4 and when strong staining when more than 4.

RETRACTED

### Statistical analysis

SPSS software (version 16.0, Chicago, IL) was used for statistical analyses. Data were presented as mean ± S.D. from at least three separate experiments. Categorical variables were compared by χ^2^ test or Fisher’s exact test. Continuous variables were compared using independent two sample *t* test. Multivariate analyses were performed by the Cox proportional hazard model. Survival curves were done by the Kaplan–Meier method (the log-rank test). All tests were two-tailed and *P*<0.05 was considered to be statistically significant.

## Results

### C14orf166 was up-regulated in human NSCLC tissues and cell lines

To investigate the protein expression of C14orf166 in NSCLCs, IHC staining was primitively used in 125 NSCLC primary tumor samples and in paired adjacent normal samples. Figure 1A shows that weak or no immunoreactivity was observed in the adjacent normal tissues; in contrast, C14orf166 protein was found to be highly expressed in both the carcinoma cell nuclei of lung adenocarcinoma and lung squamous carcinoma cells, and with the cytoplasmic reaction was occasionally displayed. According to previously mentioned standards [23], the strong staining rate of C14orf166 protein in the NSCLC group was 78.4% (98/125), while it was 11.2% (14/125) in the paired normal tissues group (*P*<0.001, Figure 1A). This discrepancy in the expression pattern of the C14orf166 protein was confirmed by Western blotting analysis (Figure 1D). Furthermore, *C14orf166* mRNA expression was analyzed by qRT-PCR in 125 cases of NSCLCs and in their paired adjacent normal tissues. We found a similar tendency of C14orf166 expression at the mRNA level (Figure 1B). The overall average expression level of C14orf166 was markedly up-regulated (3.72 times) in tumor tissues than in adjacent normal tissues (Figure 1B). Moreover, high C14orf166 expression (more than two-fold namely, log_2_ (fold change) > 1) was observed in 75.2% cases (94/125) (Figure 1B and Table 1) when compared with *C14orf166* mRNA expression in NSCLCs and those in paired adjacent normal tissues, suggesting that the overexpression of C14orf166 was a frequent event in human NSCLC.

RETRACTED

**Figure 1:** C14orf166 was frequently overexpressed in NSCLC (**A**) The expression of C14orf166 protein was assessed in normal and NSCLC tissues by IHC staining. Representative images of negative staining of C14orf166 in normal lung tissues (upper left), weak staining, and strong staining of C14orf166 in lung adenocarcinoma tissues (upper middle, upper right), weak staining, and strong staining of C14orf166 in lung squamous carcinoma tissues (lower left, lower middle). Compared with the normal lung tissues, the NSCLC tissues were detected to express more C14orf166 in the nuclei significantly (lower right). (**B**) The relative expression of *C14orf166* mRNA in 125 NSCLC patients. Data were analyzed using a −ΔΔ*C*_T_ (NSCLC/normal) approach and expressed as log_2_ fold change (−ΔΔ*C*_T_). (**C**) *C14orf166* mRNA expression in NSCLC cell lines (A549, PC-9, and HTB182) and HBE. Each sample was analyzed in triplicate, and values are expressed as levels (mean ± S.D.) relative to those in HBE cells. (**D**,**E**) Representative images for C14orf166 protein in NSCLC tissues and cell lines compared with normal lung tissues and cell lines by Western blotting, respectively. (**F**) The positive correlation between *C14orf166* mRNA levels and C14orf166 protein expression. Fold expression or fold change of *C14orf166* mRNA was shown as 2^−ΔΔ*C*^_T_, **P<0.01.

**Table 1:** Correlations between C14orf166 expression and clinicopathological variables of 125 cases of NSCLC

		C14orf166 expression		
Clinicopathological variables	*n*	Low	High	*P*
Age (years)				
≤60	67	15	52	
>60	58	16	42	0.502
Gender				
Female	32	10	22	
Male	93	21	72	0.327
Smoking history (years)				
≤10	26	9	17	
>10	99	22	77	0.193
Pathological type				
Adenocarcinoma	56	15	41	
Squamous carcinoma	69	16	53	0.643
Differentiation				
Well	54	11	43	
Moderate	43	15	28	
Poor	28	5	23	0.162
T classification				
T1	24	10	14	
T2	35	13	22	
T3	44	6	38	
T4	22	2	20	**0.006**
N classification				
N0	65	25	40	
N1	32	4	28	
N2	28	2	26	**0.001**
TNM stage				
I	33	20	13	
II	39	7	32	
III	53	4	49	**<0.001**
Chemotherapy				
No	69	7	62	
Yes	56	24	32	**<0.001**

*P*-values <0.05 are indicated in bold.

C14orf166 expression in NSCLC cell lines and HBE was also detected by qRT-PCR and Western blotting. As shown in Figure 1C,E, compared with the expression in normal cells (HBE), *C14orf166* mRNA and protein expression levels were significantly increased in human NSCLC cell lines (A549, PC-9, and HTB182).

Moreover, as Figure 1F shows, the relative expression of *C14orf166* mRNA was positively associated with the IHC staining score, which indicated that C14orf166 was up-regulated in NSCLC both transcriptionally and translationally.

RETRACTED

### Elevated C14orf166 expression was related to clinicopathologic characters in NSCLC

The association between *C14orf166* mRNA expression and the clinicopathological features of NSCLCs was explored by the χ^2^ test or by Fisher’s exact test. As summarized in Table 1, the high expression of C14orf166 was significantly associated with T classification (*P*=0.006), lymph node metastasis (*P*=0.001), TNM stage (*P*<0.001), and chemotherapy (*P*<0.001). The high C14orf166 expression rate was 68.7% in females and 77.4% in males. However, there was no significant relationship between C14orf166 expression and variables such as age (*P*=0.502), gender (*P*=0.327), smoking history (*P*=0.193), pathological type (*P*=0.643), or tumor differentiation (*P*=0.162). A subgroup analysis revealed that overexpressed C14orf166 was associated with advanced stage and with lymph node metastasis (Figure 2A,B).

**Figure 2:** C14orf166 was a promising prognostic biomarker for NSCLC (**A**) Relative *C14orf166* mRNA expression levels in NSCLC tissues at different TNM stages: I, II, and III. (**B**) Relative *C14orf166* mRNA expression level in lymph node metastases: (+) or (−) NSCLC tissues. (**C**,**D**) Survival relevance analysis of *C14orf166* mRNA expression in NSCLC patients. According to the qRT-PCR data, the expression of C14orf166 was classified into high expression (*n*=89) and low expression (*n*=31). Fold expression or fold change of *C14orf166* mRNA was shown as 2^−ΔΔ*C*^_T_.

### Overexpressed C14orf166 was associated with the poor prognosis of NSCLC

In the present study, we successfully followed up with 120 patients (loss rate is 4.0%), and the mean follow-up duration was 37.15 months (5–60 months). To assess the potential role of C14orf166 expression in NSCLC prognosis, a Kaplan–Meier survival analysis and log-rank test were performed. Expression of C14orf166 was tightly associated with survival time. The patients with overexpression of C14orf166 had much shorter overall survival time (median survival time, 32 compared with more than 60 months) (*P*<0.001, Figure 2C) and shorter disease-free survival (median survival time, 29 compared with more than 60 months) than those with low C14orf166 expression (*P*<0.001, Figure 2D).

To assess the feasibility of C14orf166 expression in predicting NSCLC prognosis, the Cox proportional hazards regression model was conducted. From multivariate survival analysis, T classification (*P*<0.001), N classification (*P*<0.001), TNM stage (*P*=0.001), chemotherapy (*P*=0.017), and C14orf166 expression (*P*<0.001) reached significance in terms of overall survival (Table 2). For the analysis of disease-free survival time, T classification (*P*=0.001), N classification (*P*<0.001), TNM stage (*P*=0.001), chemotherapy (*P*=0.043), and C14orf166 expression (*P*=0.001) reached significance in the multivariate survival analysis Cox proportional hazards regression model (Table 2).

RETRACTED

**Table 2:** Cox regression multivariate analysis of overall and disease-free survival in 120 patients with NSCLC

		Overall survival		Disease-free survival	
Variables	*n*	HR (95%CI)	*P*	HR (95%CI)	*P*
Age (years)					
≤60	64	1		1	
>60	56	1.60 (0.93–2.73)	0.089	1.45 (0.86–2.46)	0.164
Gender					
Female	30	1		1	
Male	90	0.99 (0.54–1.81)	0.978	0.96 (0.53–1.71)	0.878
Smoking history (years)					
≤10	24	1		1	
>10	96	1.50 (0.79–2.83)	0.216	1.37 (0.73–2.58)	0.331
Pathological type					
Adenocarcinoma	53	1		1	
Squamous carcinoma	67	0.84 (0.50-1.39)	0.489	0.78 (0.47-1.29)	0.330
Differentiation			0.154		0.186
Well	53	1		1	
Moderate	43	0.73 (0.37–1.43)	0.358	0.71 (0.38–1.34)	0.291
Poor	24	1.36 (0.63–2.97)	0.435	1.27 (0.57–2.78)	0.560
T classification			**<0.001**		**0.001**
T1	22	1		1	
T2	33	0.64 (0.18–2.33)	0.502	0.96 (0.28–3.31)	0.952
T3	43	2.25 (0.69–7.27)	0.177	2.59 (0.80–8.40)	0.112
T4	22	9.38 (2.48–35.54)	**0.001**	8.04 (2.09–30.98)	**0.002**
N classification			**<0.001**		**<0.001**
N0	64	1		1	
N1	30	2.52 (0.82–7.77)	0.108	2.16 (0.71–6.51)	0.173
N2	26	12.55 (3.23–48.76)	**<0.001**	9.58 (2.50–36.80)	**0.001**
TNM stage			**0.001**		**0.001**
I	32	1		1	
II	36	13.71 (3.22–58.34)	**<0.001**	12.68 (3.28–49.11)	**<0.001**
III	52	30.01 (3.92–229.59)	**0.001**	35.06 (4.74–259.31)	**<0.001**
Chemotherapy					
No	66	1		1	
Yes	54	0.44 (0.22–0.86)	**0.017**	0.50 (0.26–0.98)	**0.043**
C14orf166 expression					
Low	28	1		1	
High	92	4.88 (2.08–11.46)	**<0.001**	4.01 (1.81–8.92)	**0.001**

*P*-values <0.05 are indicated in bold.

HR, hazard ratio; CI, confidence interval.

## Discussion

As a protein located in the nucleus and in the cytoplasm, C14orf166 was found to be a transcriptional regulator related to the repression of the centrosome architecture [6] and to be a shuttling protein, playing an important role in the regulation of cellular RNA expression through the transportation of RNAs between the nucleus and the cytoplasm [10,24]. RNAs combined with the binding complex, C14orf166–DDX1–HSPC117–FAM98B, are selected to be transported and promote expression [25]. The function of C14orf166 accounts for normal RNA transcription, mRNA expression, signal transduction, and even for important cellular phenotypes such as proliferation and apoptosis [10]. The overexpression of C14orf166 has been found to contribute to oncogenesis and to invasion behaviors in a variety of tumors [19–22].

RETRACTED

The present study took the lead to report that the overexpression of C14orf166 was associated with disease progression and poor prognosis in NSCLC. First, IHC staining displayed that C14orf166 protein expression was obviously increased in NSCLC tissues, while none or few positive reactants were found in the adjacent normal tissues. Furthermore, the statistical information revealed a significant increase in C14orf166 expression in carcinoma tissues compared with adjacent normal tissues, and a similar tendency was observed by Western blotting. Second, qRT-PCR analysis also revealed that C14orf166 mRNA was overexpressed in most cases of NSCLC, which was positively associated with the IHC staining score, indicating that C14orf166 was up-regulated in NSCLC both transcriptionally and translationally, which was in accordance with the function of C14orf166. Moreover, we found that C14orf166 was constantly up-regulated in NSCLC cell lines. These results agree with our previous study of C14orf166 in esophagus squamous cell carcinoma [18], as well as in other previous studies [22,26].

The data in the present study also showed that C14orf166 may be a promising prognostic predictor of NSCLC. First, we explored the potential correlation between *C14orf166* mRNA expression and the various clinicopathological characteristics of NSCLC patients, and we found that the increased expression of C14orf166 was nonsignificant in terms of age, gender, smoking history, and even tumor differentiation, but the study revealed a strong relationship with T stage, lymph node involvement, TNM stage and chemotherapy. It is worth mentioning that the expression of C14orf166 was undifferentiated in lung squamous carcinoma tissues and in lung adenocarcinoma lesions. Our data indicated that despite the tumor differentiation and pathological type, the higher expression of C14orf166 advanced the tumor progression, which is consistent with research in pancreatic cancer [21]. Lymph node involvement is an indicator frequently used for disease condition evaluation as well as for outcome prediction in NSCLC, which is consistent with our present study. The patients with elevated expression of C14orf166 had significantly associated with shorter overall and disease-free survival times. In addition to T stage, N stage, TNM stage, and chemotherapy, our data showed that C14orf166 expression was also an independent prognostic predicator in NSCLC patients. As an adjuvant therapy, chemotherapy is used clinically to improve prognosis in NSCLC patients, and our information also displayed that the patients with increased C14orf166 expression tended to undertake chemotherapy, which can be explained by the high expression of C14orf166 that was significantly associated with the advanced TNM stage. The majority of patients undergoing chemotherapy experienced a high frequency of severe side effects; therefore, our present study on C14orf166 may benefit clinical decision-making in NSCLC patients. Though a recent study has explored the feasibility of detected C14orf166 in blood samples [20], further validation investigations are urgently needed to discover its role as a serum biomarker for early diagnosis and as a target for therapy design.

RETRACTED

Dysfunction of signal pathways has been reported to be involved in tumor initiation as well as in progression for their crucial role associated with cellular function, such as proliferation, differentiation, survival, and apoptosis [27–30]. Consistent with other studies, our results implied that C14orf166 might participate in oncogenesis and tumor progression in NSCLC and that it might be attributed to the function of C14orf166 in cell division and signal transduction, in addition to its regulatory role in mRNA expression. It has been demonstrated that C14orf166 is associated with ninein in the centrosomes during cell division [31]. Howng et al.’s [32] research also confirms that C14orf166 may be involved and restricted to ninein phosphorylation during the cell cycle by co-operating with GSK-3β, which is thought to account for the formation and development of brain tumors. As an evolutionarily conserved serine/threonine kinase, GSK-3β phosphorylates β-catenin, which induces its degradation through ubiquitination and proteasomal activation in cytosol. It has been generally believed that abnormal GSK-3β-mediated functions are associated with carcinogenesis [33]. Excessive GSK-3β function, which is frequently observed in tumor initiation, promotes progression and contributes to drug resistance by harassing signaling pathways including the Wnt/β-catenin, PI3K-AKT-mTOR, and JAK2/STAT3 signaling pathways [34–36]. Aberrant β-catenin degradation by GSK-3β can promote lung carcinoma cells metastasis and spread [37–39]. The inhibition of GSK-3β induces β-catenin accumulation and plays a vital role in chemical agent-induced growth inhibition and apoptosis in lung cancer cells, such as tivantinib and dihydroartemisinin [40,41]. The disordered intracellular JAK2/STAT3 signaling pathway is frequent in many carcinomas and is related to malignant features; therefore, blocking of this pathway can help decrease tumor burden and to improve chemosensitivity. The inhibition of GSK-3β is crucial for xanthation to exert its anticancer properties in NSCLC, and the restraint of inherent activation of STAT3 enhances this function [42]. C14orf166 has been found to participate in the development of cervical cancer, which is thought to be involved in the abnormal JAK2/STAT3 pathway [22]. Along with the acylglycerol kinase, C14orf166 is identified as a JH2-interacting protein, which consecutively activates the JAK2/STAT3 signaling pathway to promote esophageal squamous cell generation and to enhance the cancer stem cell population [43]. Although our present study cannot reveal the innermost mechanism in NSCLC, the potential interpretation might be the exceptional signaling pathway, which is partly a consequence of the interaction of overexpressed C14orf166 and GSK-3β.

RETRACTED

In conclusion, C14orf166 is up-regulated in NSCLC and is significantly correlated with T stage, N stage, TNM stage, chemotherapy, and overall and disease-free survival. The high expression of C14orf166 is significantly associated with a poor prognosis in advanced stage and in lymph node metastasis patients with NSCLC. C14orf166 is an independent prognostic biomarker for NSCLC patients, which may provide a wider perspective on NSCLC intervention, prevention, and treatment. Though these preliminary results show the potential role of C14orf166 in NSCLC, the underlying mechanism of C14orf166 in regulating oncogenesis, progression, metastasis, and prognosis still requires further investigation.

## Abbreviations

C14orf166: chromosome 14 ORF 166
GAPDH: glyceraldehyde-3-phosphate dehydrogenase
GSK-3β: Glycogen synthase kinase-3β
HBE: human bronchial epithelial cell
HRP: horseradish peroxidase
IHC: immunohistochemistry
JAK: Janus kinase
NSCLC: non-small-cell lung cancer
PI3K-AKT-mTOR: phosphatidylinositol-3-kinase-serine/threonine kinase-mammalian target of rapamycin
qRT-PCR: quantitative real-time PCR
RIPA: radio immunoprecipitation assay
STAT3: signal transducer and activator of transcription 3
TNM: Tumor Node Metastasis
UICC: Union for International Cancer Control
